RETRACTED

# The influence of environmental diplomacy, economic determinants and renewable energy consumption on environmental degradation: Empirical evidence of G20 countries

**DOI:** 10.1371/journal.pone.0300921

**Published:** 2024-03-25

**Authors:** Muhammad Rizwanullah, Jian Shi, Muhammad Nasrullah, Xue Zhou

**Affiliations:** 1 School of Public Administration, Xiangtan University, Xiangtan, 411105, P.R China; 2 South Asia Research Centre Xiangtan University, Xiangtan, 411105, P.R China; 3 School of Marxism, Southwestern University of Finance and Economics, Chengdu, P.R China; Hong Kong Shue Yan University, HONG KONG

## Abstract

This study examines how various environmental and economic variables contribute to environmental degradation. Industrialization, trade openness, and foreign direct investment are among the variables, as are environmental diplomacy, environmental diplomacy secure, and renewable energy consumption. Therefore, the data covers the years 1991–2020, and our sample includes all 19 countries and two groups (the European Union and the African Union). The research used the Pesaran CD test to determine cross-section dependency, CIPS and CADF test to determine stationarity, the Wald test for hetrodcedasasticity and the Wooldridge test for autocorrelation; therefore, VIF for multicollinearity, Durbin and Hausman to analyze the endogeneity. It also employed Westerlund’s cointegration test to ensure cross-sectional dependence, Wald test for group-wise heteroscedasticity, Wooldridge test for autocorrelation, VIF for multicollinearity, and Durbin and Hausman for endogeneity. The two-step system generalized method of moments (GMM) is used to estimate the results and confirm the relationship between independent variables (Industrialization, trade openness, FDI, environmental diplomacy, secure environmental diplomacy, and renewable energy) and dependent variables (Environmental Degradation) in G20 countries. Therefore, Industrialization, trade openness, foreign direct investment, ecological diplomacy, and renewable energy consumption significantly impact ecological degradation. Environmental diplomacy is crucial to combat degradation and stimulate global collaboration. G20 nations enact strict environmental restrictions to tackle climate change and encourage economic growth.

## Introduction

Over the past years, environmental issues like deforestation, global warming, loss of biodiversity and pollution have alarmingly increased across the globe [1,2]. The world has adopted diplomacy to address situational environmental challenges that are interdependent on one another [3]. Environmental diplomacy is often the use of diplomatic strategies and conferences to mitigate or control environmental issues that cross borders. The phenomenon has become necessary when discussing the cooperation of the countries [4,5]. International cooperation is especially relevant among the members of the G20 group, which includes major economies, the effects of whose growth have considerable environmental impacts. In a demonstration of their intention to mediate, countries engage in treaties at various levels, bilateral, multilateral, and global [6–8]. They have broad environmental implications as industrial and commercial ties increase worldwide because of globalization, such as industrialization, trade openness, FDI, and energy consumption. This has immensely contributed to the increase in greenhouse gas emissions, especially the rise in massive quantities of carbon dioxide [9,10].

RETRACTED

Rapid ecosystem damage continues to be witnessed in addition to widespread climate change due to this increased rate [11]. The relationship between economic activity, environmental sustainability, and diplomacy has propelled environmental diplomacy as a necessary tool for ensuring environmental protection [12,13]. Industrialization, as one of the key sources of economic growth, is responsible for environmental pollution [14,15]. Global trade promotes economic integration but inadvertently stimulates polluting industries and processes. Sustainable responses on a global scale require a grasp of industrialization, trade openness, and environmental diplomacy. Foreign Direct Investment (FDI) has increased both advantages and disadvantages.

On one side, it represents technological innovativeness, and on the other–ecological awareness [16]. It provides an incentive arrangement that promotes responsive investments and mitigates the negative environmental consequences of FDI [17,18]. The energy sector has revitalized industrialization and economic growth and remains very significant in the factor of environmental degradation [19]. Countries must make use of sustainable and renewable sources of insecurity and environmental hazards. The transition to sustainable energy is often amicably achieved through negotiation and agreement, as well as diplomatic collaborations that encourage the development and implementation of renewable energy sources [20,21]. To understand the bigger purpose of minimizing ecological degradation, one might have to be cognizant of the role played by environmental diplomacy in promoting renewable energy sources and promoting the security of energy [22]. Coastal and Land-based pollution and the destruction of forests and soil were causes of the increase in CO2 emissions, one of the greenhouse gases [23]. CO2 consequences related to climate change further need a global structure led by the interwoven relationship between environment diplomacy and nations to find solutions, establish measures, set reduction targets, and promote eco-friendly practices to stop CO2 pollution [24].

RETRACTED

The purpose of this research is to investigate the intricate relations and causal chains between industrialization, trade openness, foreign direct investment (FDI), environmental diplomacy, secure environmental diplomacy, renewable energy consumption, and environmental degradation, with a particular focus on carbon dioxide (CO2) emissions in environmental diplomacy. The objectives of this study are to assess the diplomatic history of environmental policies among G20 countries, analyze their impacts, and determine the consequences of economic development on ecological sustainability. So, this study contributes to understanding global attempts to prevent negative changes occurring in the natural environment. The aim is to provide evidence-based advice to policymakers, diplomats, and environmental activists to strengthen international cooperation and initiatives targeting climate change and ecological sustainability. Alternatively, the main objective is to provide evidence-based guidance to policymakers, diplomats, and environmentalists, which aims to improve international agencies and interventions to address climate change.

### Objective

The following are the objectives:

- To analyze the effect of Environmental Factors on the ED.
- To analyze the effect of Economic Factors on the ED.

### Literature review

This literature offers various points of view regarding the intricate relations between economic activity, diplomatic options, and environmental preservation. This literature review critically assesses the intricate co-variations between industrialization, trade openness, FDI, Renewable energy consumption, and ecological degradation in the case of the G 20 countries. This study’s objective essentially lies in analyzing the evolution of environmental diplomacy on international economic exchanges over time by analyzing information from different sources. Key concepts, information, and policy frameworks, which are intricately linked, forming a vital aspect of how these interrelated factors impact the environment and affect international partnerships and environmental sustainability, are investigated in the study.

### Industrialization and environmental degradation

Industrialization brings economies from agriculture based on products and implements mechanized manufacturing and technological progress that help solidify the economy and have favorable effects on living standards [25]. At the same time, it demonstrates the impact of environmental issues such as pollution, deforestation, the destruction of habitats, and climate change. According to Nwafor [26], there must be effective ways to balance economic development and ecological sustainability in favor of cleaner technologies, sustainable practices, and implementation measures accompanied by strict environmental regulations. In the past, everything about industrialization and ecological degradation was seen as expansive literature related to the relationship between industrialization and environmental degradation. Industrialization in 37 African countries has only led to more degradation because of industrialization in the 10 to 30 percent quantiles. Still, industrialization has led to less environmental degradation in the 40 to 90 percent quantiles. To combat this, manufacturing firms should adopt greener technologies and enforce environmental regulations to contribute to sustainable development and environmental protection [27]. According to Opoku [27], industrialization and foreign direct investment have been found to have significant environmental impacts in 36 African countries from 1980 to 2014. While industrialization’s effect on the environment is generally insignificant, the impact of foreign direct investment is largely significant. This study highlights the need for policy implications in addressing environmental degradation.

RETRACTED

Similarly, Nasrullah [28] demonstrated that industrialization is crucial for economic growth and employment generation but also poses harmful environmental effects. In China, 83 cities have PM2.5 levels greater than or equal to 35, causing significant pollution. This silent killer affects air, water, and food, affecting everyone’s lives. Despite economic advancements and power, pollution remains a constant threat, affecting the environment and hindering economic growth. Therefore, it is essential to address pollution and promote sustainable development. Besides, CO2 emission refers to the air pollutant level in India, and the study’s research analyses India’s industrial developpment, economic growth, fossil fuel energy output, financial development and globalization as assessed by the CO2 emission effects. It uncovers a long-term correlation between CO2 emissions and the other factors, which are industrialization and economic growth, positively impacting CO2 emissions. From these findings, policymakers must improve economic development while ensuring that a negligible amount of environmental depletion occurs [29].

Furthermore, according to research Patnaik [30], industrialization has led to economic prosperity, increased population, and urbanization, putting environmental impacts at risk. Transitioning industries into eco-industrial networks through green approaches can preserve natural resources and enhance the economy. A study on industrial pollution in Puducherry reveals severe impacts and root causes, highlighting the need for sustainable solutions to curb pollution and improve environmental sustainability in the region. This study’s hypotheses are derived from the previous literature review:

***H1*:** *Industrialization has significant impact on the Environmental Degradation*.*\*

RETRACTED

### Trade openness and environmental degradation

Trade openness refers to a nation’s market accessibility for international trade, reducing barriers to moving goods and services [31]. Globalization, characterized by reduced tariffs, fewer import and export restrictions, and enhanced economic integration, is often evaluated regarding environmental degradation and its effects on the natural environment [32]. Previously, much literature was available on the relationship between trade openness and environmental degradation. According to the study [33], the impact of industrial expansion and trade openness on environmental degradation was investigated in 16 Asian economies from 1992 to 2020 using panel data. The results are obtained using a panel unit root test followed by the Panel ARDL technique. The unit root test results suggest using the ARDL approach, which estimates both short- and long-term effects. The research information on CO2 emissions indicates that the increase in CO2 emissions in Asian countries is due to the increase in population and the value additions regarding the industries in these areas.

Conversely, trade openness, government expenditure, and GDP have a mitigating effect on CO2 emissions. According to the researcher Nasrullah [21], trade openness plays a crucial role in China’s economic development and poses environmental challenges. This study examines the impact of trade liberalization on environmental pollution in China, focusing on its eastern, central, and western regions. Findings indicate that trade openness correlates negatively with industrial emissions of CO2 and positively with industrial wastewater emissions in an inverted “N” and “U” pattern.

The effects of carbon dioxide emissions from Sub-Saharan Africa (SSA) on human health and climate change are investigated by Rizwanullah et al [13]. This study examines the relationship between trade openness, foreign direct investment (FDI), and environmental deterioration in Sub-Saharan Africa (SSA) using a time series dataset that spans 1975 to 2020. Research makes use of quadratic modelling and tipping points within the EKC framework. Both trade openness and foreign direct investment (FDI) did not correlate with the environmental Kuznets curve (EKC). Implications in the long run grow, while those in the near run diminish. The relationship between trade openness and foreign direct investment is U-shaped. While trade openness and FDI decrease in the short run, they increase in the long run. The research previously supported the halo effect theory but has now shifted its focus to the pollution haven theory. Similarly, this research explores the association between trade openness and CO emissions in African countries. It helps to uphold the hypothesis of a “pollution haven”, and the conclusion affirms that trade-free with CO2 emission tends to increase CO2 emission. However, the elasticity also differs significantly across measures. In addition, a “scale” effect between higher quintiles and the 90^th^ percentile can be observed as trade openness increases in some quintiles but decreases at the 90^th^ percentile [34].

RETRACTED

Furthermore, according to the researcher [35], the debate discussed the relationship between international trade and environmental outcomes. Theoretical work has proposed various hypotheses, but empirical verification still needs to be improved. The study focuses on the effects of Sub-Saharan Africa (SSA) carbon dioxide emissions on human health and climate change. Using a dynamic autoregressive distributed lag (ARDL) simulation architecture, the study zeroes in on South Africa and examines time series data from 1960 to 2020. Although there is a positive effect in the short run, the research shows that trade openness negatively affects environmental quality in the long run. The study also verifies the existence of an EKC hypothesis, which states that CO₂ emissions are increased by the scale effect and decreased by the method effect. Energy consumption, FDI, and industrial value-added are some of the factors that contribute to environmental degradation, whereas technical innovation improves environmental quality. This study’s hypotheses are derived from the previous literature review:

***H2*:** *Trade Openness has significant impact on the Environmental Degradation*.

### Foreign direct investment and environmental degradation

Foreign Direct Investment (FDI) is a corporate-driven phenomenon whereby a company or individual from a country invests in business activities in another country’s location. However, the meaning of FDI in environmental degradation is based on the nature and operations of the investing companies and the country’s environmental regulations and policies [21]. This study A’yun [36] evaluates the relationship between ecological capital, economic growth, trade openness, and global warming in 10 ASEAN nations. The primary focus is on trade liberalization and economic development, which cause changes in carbon dioxide emissions. Based on panel data analysis, the study’s analyses establish a substantial negative relationship between economic growth and carbon dioxide emissions. Imports are not statistically related to carbon dioxide emissions in the first stage; the second stage finds that exports and foreign direct investment have positive and statistically significant impacts on carbon dioxide emissions. Research ends with the observation that in ASEAN states carbon emissions should be reduced through regulation based on environmentally friendly technologies. From this point of view, the factors that cause environmental degradation in some OIC member countries can be determined by knowledge of foreign direct investment (FDI), institution effectiveness, and technological advancement [37]. Between 2000 and 2022, the panel data were studies of the lowly middle-income countries belonging to the following nations. These findings suggest that sustained scientific development significantly scales down the ecological footprint in lower-middle-income economies. Still, FDI is negative for inducing this impact on a large scale. This indicates an increase in middle-income countries institutional Performance, and production on that account decreases. The openness of trade has a positive and large impact on the ecological footprint, even though the level of per capita GDP does not influence this factor in any way.

RETRACTED

Likewise, this study investigated the effect of environmental degradation on foreign direct investment (FDI) in ASEAN+3 countries. Based on the study, inflation has a short-term impact on FDI. On the contrary, environmental deterioration, infrastructure, and corruption have long-included effects. In efforts to boost their foreign direct investment (FDI), the findings suggest that governments should implement infrastructure development, curb corruption and inflation, and provide environmental incentives [38,39] present a study that shows FDI affected the environmental quality of nations in CEE between 1995 and 2014. This study deals with FDI, GDP growth, energy consumption, and carbon dioxide emission, all conducted through panel econometric methods. As the analysis of the role of FDI in the effects of environmental quality suggests, the result looks to have a reverse U-shaped kind of effect that is nonlinear. Sustainable development is assumed to significantly impact the improvement of environmental performance due to economic growth, as suggested by the research. The research area considers issues of FDI, and sustainable development and issues related to energy and environmental policy in CEE. Besides, financial development and foreign direct investments (FDI), under the supposition of eighty-three developing and developed countries between 2000 and 2017, are studied in this paper to determine the effects on carbon emission. It reveals that the negative impacts of financial depth in institutions are lower compared to developed economies, while it negatively influences CO2 intensity in developing economies. The qualification of inward FDI stock affects CO2 intensity in developing countries [21].

RETRACTED

Furthermore, Nasrullah [21] stated that the ecosystems of the BRICS countries are deteriorating due to FDI. According to the study, foreign direct investment (FDI) and GDP considerably lower CO2 emissions in these nations. The data bear out neither the pollution haven hypothesis nor the environmental Kuznets curve idea. The report suggests employing cleaner technology, encouraging foreign direct investment (FDI) that prioritizes environmental awareness, enacting legislation to combat climate change, and delegating environmental procedures effectively. This study’s hypotheses are derived from the previous literature review:

*H3*: *Foreign Direct Investment has significant impact on the Environmental Degradation*.

### Environmental diplomacy and environmental degradation

Environmental diplomacy involves diplomatic strategies, negotiations, and global collaboration to tackle cross-border environmental issues and advance sustainable resolutions [19]. Environmental diplomacy promotes international cooperation in addressing environmental degradation, including pollution, biodiversity loss, climate change, and other related concerns [40]. Previously, much literature was available on the association between environmental diplomacy and environmental degradation. International environmental agreements, including environmental diplomacy, significantly mitigate carbon dioxide emissions, as covered by Khan and Hou [41]. Such effects are induced in the present day, such as an elevation of the use of eco-friendly energy, capital formation, and economic growth, which are high-quality declining factors. Although the study showed that the fear of strong diplomatic contacts and reciprocity of the commitment is essential, further diplomacy may increase CO2 emissions. It has been demonstrated that there has been a temporary reduction in emissions in developing nations due to environmental diplomacy, which is one of the aspects of international diplomacy [21]. Nevertheless, these studies are all-inclusive, and there are first-hand findings that show that governments often do not accept the treaties by going ahead and negating the treaties they carry out, leading to increased CO2 emissions.

RETRACTED

Based on the study, the countries should not sign treaties annually but have the treaties proved, and authorities should concentrate on fulfilling their duties. This has led to the belief that this would not significantly impact climate change. Additionally, as Nasrullah [21] argued, environmental diplomacy is an essential feature in this type of international cooperation to tackle environmental issues. The conflicts between developed and underdeveloped countries, the unpredictability of predicting environmental threats, and the inability of the United Nations to resist environmental threats have each slowed down the current new treaty-making effort of even the Earth Summit in 1992 in Brazil. Sustainable Development is proposed by a distinguished environmental diplomat, Lawrence Susskind, who suggests nearly self-enforcing agreements that cannot threaten the nation’s sovereignty while ensuring compliance and future new institutional arrangements for sustainable Development. This study’s hypotheses are derived from the previous literature review:

*H4*: *Environmental Diplomacy has significantly impact on the environmental degradation*.

### Environmental diplomacy secure and environmental degradation

The phrase ‘primary energy supply’ refers to total energy amount produced naturally without any conversion or formulation processes before using [42]. Energy availability is measured in physical units such as those measured in joules or British thermal units, which can be used to quantify the amount of energy available for consumption [43]. The basis for environmental degradation is ensured by primary energy supply through different ways of sourcing this energy, which in turn, it has been both in terms of the methods and sources, could result to environmental impacts [44]. For environmental diplomacy fragile and pollution particularly, many studies had considered the previous research that generated large amounts of literature had been written about the relation of environmental diplomacy fragile and pollution.

Zakari et al [45] demonstrated that, factors such as primary energy supply and green financing influenced the performance environmental and Japan and China over the period of 2010–2020. Consistent with the results, primary energy supply promotes environmental performance, but the latter also supports environmental sustainability because of the reduction pollutant pressure. The research state that grants and subsidy therefore should be introduced to help develop the green energy system. China’s environment has been deteriorating at an alarming rate accordingly to the experts Butt [46] because of its rising consumption of energy and extensive utilization of fossil fuels. This has led to a domino effect in terms of environmental problems whereby the institution has contaminated both air and water as well as soil erosion. To address these challenges, China must take steps aimed at reducing its energy consumption and fostering a culture energy conservation while transitioning to cleaner, more sustainable energy. In the research, it is stated that the main energy supply has the strongest impact on the ecological footprint, while consuming of energy and foreign trade cause less influences. A significant area that policy makers should pay consideration to energy is the transportation and industrial sectors. Also, as it is indicated by Deka [47], reliable and stable energy provision lies at the core of the European Union’s unimpeded economic growth because such energy is fundamental in it. To examine the impact of the primary energy supply on economic growth in the EU, the framework was employing panel data of 27 EU states for the period from 1990 to 2019. The findings showed that among the 27 European Union member states, carbon emissions, renewable energy, capital, effective capital, and population size positively affect GDP. While the DOLS method had a notable positive impact on GDP, the primary energy supply had the opposite effect. This study’s hypotheses are derived from the previous literature review:

***H5*:** *Environmental Diplomacy secure has significant impact on the Environmental Degradation*.

RETRACTED

#### Renewable energy consumption and environmental degradation

Renewable energy consumption involves using energy from sources that naturally replenish themselves within a timeframe relevant to human activities [16]. The sources encompass solar, wind, hydropower, geothermal, and biomass [48]. Renewable energy consumption is closely linked to environmental sustainability as it involves transitioning away from finite and environmentally harmful fossil fuels, thereby helping mitigate environmental degradation [11]. Previously, much literature was available on the association between renewable energy consumption and environmental degradation. The research explored the impact of GDP growth, technological innovation, and energy sources on CO2 emissions in Spain, aiming to develop an SDG framework for other EU nations. The relations that are observed here are based on data from IDB (1980–2018). According to the results, an increase in shocks from renewable energy consumption is associated with the improvement of environmental quality, while the increase of shocks in technological innovation leads to fewer CO2 emissions [49]. On the other hand, positive disturbances in energy utilization raise CO2 hits. The policy implications of this study for Spain and the rest of the neighbors are apparent.

RETRACTED

As stated by Ayobamiji [50], renewable energy, a non- carbohydrate source of energy, can as well contributes positively towards sustainable development and environmental quality. Activities that use the renewable energy sources in Vietnam may be influenced by the political disequilibrium, economic development, and globalization. Political risk and environmental rebound have a negative effect on economic development, leading to the flourishing of renewable energy both in the medium and long term as found by the study. Based on the results of this study, the economic globalization will also be correlated with the renewable energy in Vietnam FDI, transfer of technology, and capital information are expected to facilitate the use of the renewable energy in Vietnam.

Likewise, Byaro [51] showcase how, between 2000–2020, environmental degradation, renewable energy use, and natural resources depletion interplayed in 48 nations of sub-Saharan Africa. As suggested, the revealed results bear out that affected by more intense natural resource depletion countries are prone to be correlated with the environmental depletion, while less depletion affected countries will be vulnerable to be connected to the negative environmental effect. Industrialization and commercialization plus economic development in a long run narrow the menace of the environmental threats; however, the rise of the renewable energy forms reduce the danger to a great level. Policy makers should therefore prioritize on poverty reduction and the growing of other renewable energy sources as the best way of improving the stability and the security of its geopolitical position. Additionally, the research indicates that sustaining the SDGs requires the continued utilization of renewable energy resources. Money and politics play part in the use of renewable energy as a regular source of energy. This study suggests that risk management for these risks is one of the mitigation techniques as shown in ASEAN’s plan to mitigate its ecological footprint (EF) and achievement of SDGs. The fact that using renewable energy is associated with lower EF demonstrates the significance of managing political and financial risks for long-term sustainability. This study’s hypotheses are derived from the previous literature review:

***H6*:** *Renewable energy consumption has significant impact on the Environmental Degradation*.

## Methodology

### Conceptual framework

A thorough review of the relevant empirical literature enabled the conceptual framework’s development. This research examines how the environmental degradation of G20 countries has an effect due to industrialization, trade openness, FDI, environmental diplomacy, environmental diplomacy secure, and renewable energy consumption. **Fig 1** displays the entire Research Model.

RETRACTED

**Fig 1:** Research model.

### Data

This study is a quantitative type of research, which seeks to explain relationships among variables since the primary objective that we examine how industrialization, trade openness, FDI, environmental diplomacy, security, and renewable energy consumption affect environmental degradation. Using panel data, our sample comprises all G20 countries, and our data ranges from 1991 to 2020. The data for all variables comes from the World Bank’s Global Financial Development Database (GFDD) and IMF. The independent variables include industrialization, trade openness, FDI, environmental diplomacy, security, and renewable energy consumption, while the dependent variable is environmental degradation. Table 1 lists the variables used.

**Table 1:** Definition of variables.

Variables	Code	Measurement
Environmental Degradation	ED	CO2 Emissions (Metric tons per Capita)
Industrialization	IND	Industry (Including Construction), Value added (Constant 2015 US$)
Trade Openness	TO	Imports of goods and services (%of GDP)
Foreign Direct Investments	FDI	Net Flows (%GDP)
Environmental Diplomacy	ED	Cumulative number of treaties
Environmental Diplomacy Secure	EDS	Total % of primary energy supply
Renewable Energy Consumption	REC	Total % of final energy consumption

**Data Sources:** World Band and Global Financial Development Database.

### Analysis techniques

First, we implement the cross-section dependency test (CD) by Pesaran [52] by performing Friedman statistics to assess the panel of countries’ cross-section dependency. Additionally, the panel unit root tests are performed before the main estimations, as the tests are essential to help check and see whether the variables are non-stationary. The other two tests are CIPS and CADF [56] tests, which are used to check the stationarity of selected data. Based on econometric theory, the test for this study was undoubtedly a cointegration test. For cointegration statistics, the present investigation used Westerlund’s [53].

Cointegration test to determine cointegration. This is because traditional cointegration tests for panels fail to consider cross-sectional dependence in the elements of a variable, and hence, the wrong inferences are drawn. The present research employed the Wald test to determine the group-wise heteroscedasticity, and the Wooldridge test revealed. Next, VIF was utilized for the multicollinearity and Durbin-Hausman tests to evaluate the second assumption. This study was used to examine the short and long-term relationship between our research variables, which produces consistent results even with heterogeneity and CD [54], second-generation unit root test for panel data and Westerlund for cointegration test. There are two types of GMM estimators: the Arellano Bond difference GMM, introduced by Arellano and Bond in 1991, and the Arellano-Bover/Blundell-Bond system GMM estimators, introduced by Arellano and Bover in 1995 and Blundell and Bond in 1998. GMM controls for endogeneity, heterogeneity, unobserved panel, autocorrelation, omitted variable bias, and measurement errors, according to Nasrullah [21] claims that the unit root property biases the difference GMM estimator, but System GMM produces more accurate results. The differenced GMM technique removes fixed effects and differentiates all regressors to fix endogeneity.

RETRACTED

Consequently, Ullah [55] highlight the necessity to rectify the first difference transformation, as it omits the preceding observation from the present one, leading to more substantial gaps in data loss. Predictably, this has a particular impact on the anticipated result. System GMM applies fixed effects and uncorrelated (exogenous) modifications to the instruments. Incorporating additional instruments to account for endogeneity and the lagged dependent variable, among other endogenous variables, significantly improves efficiency. In addition, unlike Differenced GMM, System GMM calculates the average of all forthcoming observations of the given variables by subtracting it from the current one [56]. Consequently, this research investigated the relationship between the dependent and explanatory variables using a two-step System GMM. Diagnostic tests are unnecessary due to the inherent ability of GMM to account for endogeneity, autocorrelation, and heteroscedasticity. Nevertheless, we ensured that the data we collected was endogenous. Consequently, two-step systems GMM emerges as the most optimal approach to identify and rectify the endogeneity issue. The graphical abstract or the road map of the study are shown in **Fig 2.**

**Fig 2:** Methodology road map.

The present scenario utilizes the subsequent empirical model:

$$L_{n}({ED}_{t-1})=\beta_{0}+\beta_{1}L_{n}({IND}_{t-1})+\beta_{2}Ln({TO}_{t-1})+\beta_{3}Ln({FDI}_{t-i})+\beta_{4}Ln({ED}_{t-1})+\beta_{5}Ln({EDS}_{t-1})+\beta_{5}Ln({REC}_{t-1})+\epsilon it$$ (1)

The following is a general Model for a GMM estimator in a dynamic panel data model:

$${Ln(ED)}_{ct}=\beta_{o}+\gamma {\left(LnED\right)}_{ct-1}+\beta_{1}{\left(LnIND\right)}_{ct}+\beta_{2}{\left(LnTO\right)}_{ct}+\beta_{3}({LnFDI)}_{ct}+\beta_{4}({LnED)}_{ct}+\beta_{5}({LnEDS)}_{ct}+\beta_{6}({LnREC)}_{ct}+\mu_{ct}$$ (2)

***Note*:** *β*_0_ is the “Constant-term”, β is “Coefficients of the explanatory variables” Where Edct, INDict, Toct FDIct, Edct, EDSct and RECct is the explanatory variables for model and where u is an i.i.d. error term.

RETRACTED

## Results and discussion

### Results

#### Descriptive statistics

Descriptive statistics results demonstrated in Table 2, each variable possesses a positive Skewness value greater than zero. Consequently, every variable is represented by right-word Skewness indicators. Furthermore, all variable distributions exhibit fat-tailed behavior since the kurtosis exceeds zero. Skewness and kurtosis tests independently determined that all variables deviated from normality. Following that, the Jarque-Bera test validated the results.

**Table 2:** Descriptive statistics.

	Ln (Co2)	Ln (IND)	Ln (TO)	Ln (FDI)	Ln (ED)	Ln (EDS)	Ln (REC)
Mean	1.833	23.975	3.700	-0.123	5.991	1.759	1.982
Median	2.021	24.755	3.735	0.125	6.116	2.010	2.270
Maximum	3.019	29.466	5.339	2.544	6.507	3.844	4.068
Minimum	-0.371	17.442	1.805	-8.983	4.852	-4.605	-4.605
Std. Dev.	0.780	2.623	0.600	1.384	0.454	1.631	1.665
Skewness	0.709	0.895	0.230	1.541	0.860	2.142	2.330
Kurtosis	2.844	3.242	3.068	8.025	2.755	8.677	9.607
Jarque-Bera	47.552	76.325	57.073	812.276	70.602	1182	1527
Sum	1028	13450	2076	-69	3361	987	1112
Sum Sq. Dev.	341	3853	201	1073	116	1489	1553
Observations	561	561	561	561	561	561	561

#### Correlation matrix

Table 3 shows the results of the variables correlation matrix. The findings revealed an inverse relationship between environmental degradation and industrialization, trade openness, secure environment diplomacy, and renewable energy consumption in G20 countries. Moreover, the statistics show low, medium, and significant correlations between the various indicators.

**Table 3:** Correlation matrix.

	Ln (Co2)	Ln (IND)	Ln (TO)	Ln (FDI)	Ln (ED)	Ln (EDS)	Ln (REC)
Ln (Co2)	1						
Ln (IND)	-0.055	1					
Ln (TO)	-0.012	-0.156	1				
Ln (FDI)	0.367	-0.048	-0.023	1			
Ln (ED)	0.089	-0.004	0.091	0.332	1		
Ln (EDS)	-0.543	-0.004	0.108	0.023	0.067	1	
Ln (REC)	-0.527	-0.182	0.124	0.030	0.063	0.030	1

#### Cross-sectional dependency test

It is essential to determine whether the research variables exhibit cross-sectional dependence or independence. The outcomes of the cross-sectional dependence (CD) test are presented in Table 4.

**Table 4:** Cross-sectional dependency test.

Test	Statistic	Decision
Pesaran	4.725	Cross-sectional dependency
Friedman	19.861	Cross-sectional dependency

#### Unit root test

Prior to estimating the model, it is essential to ascertain whether all variables exhibit stationarity, as variables that lack stationarity can introduce misleading complications into regression analysis. The initial stage in panel data analysis is determining whether to employ first- or second-generation unit root tests. The information necessary to validate the presence of cross-sectional dependence is presented in Table 4. The results obtained from the second-generation CADF and CIPS tests, which examine stationary variables, will be more precise. Table 5 presents the outcomes of evaluations conducted using CIPS and CADF, two second-generation unit roots. The first difference, leads to rejecting the null hypothesis regarding unit roots. Due to these findings, the variables will maintain stationary at their first difference I (1).

RETRACTED

**Table 5:** Second generation unit root test.

Variable	Test	At level	At first difference
Ln (CO2)	CIPS	0.947 (*)	0.125 (***)
	CADF	0.188 (no)	0.135 (***)
Ln (IND)	CIPS	0.796 (no)	0.097 (**)
	CADF	0.126 (no)	0.303 (***)
Ln (TO)	CIPS	0.582 (no)	0.832 (***)
	CADF	0.775 (no)	0.924 (***)
Ln (FDI)	CIPS	1.216 (no)	0.182 (***)
	CADF	0.933 (*)	0.175 (***)
Ln (ED)	CIPS	0.136 (no)	0.035 (**)
	CADF	0.752 (no)	0.522 (***)
Ln (EDS)	CIPS	0.546 (no)	0.052 (**)
	CADF	0.683 (no)	0.199 (***)
Ln (REC)	CIPS	0.023 (no)	0.100 (***)
	CADF	0.123 (no)	0.099 (***)

**Notes:** CO2 = Carbon Dioxide Emissions, IND = Industrialization, TO = Trade Openness, FDI = Foreign Direct Investment, ED = Environmental Diplomacy, EDS = Environmental Diplomacy Secure, REC = Renewable Energy Consumption. The sign of ***, **, and * indicates that significant level at 1%, 5%, and 10%.

#### Cointegration test

According to econometric theory, this research certainly employed a cointegration test. The present investigation employed Westerlund [53] cointegration test to ascertain cointegration. This is because conventional panel cointegration tests fail to consider cross-sectional dependence among variables, which leads to erroneous conclusions. It examines whether the panels are interdependent in terms of cross-section. Table 6 displays the results of the Westerlund cointegration test. Based on the critical values supplied by the bootstrapped sturdy, three out of four tests disprove the null hypothesis, as shown in Table 6, which presents the results of the Westerlund test. These statistics indicate that the determinants have a long-lasting relationship. Testing for endogeneity was required before proceeding. Table 7 presents the results of the endogeneity test.

**Table 6:** Wester lund for panel cointegration test.

Statistic	Ga	Gt	Pt	Pa
Value (p-value)	-9.920 [0.021]	-8.317 * [0.000]	-8.917* [0.000]	-11.382 [0.018]

RETRACTED

**Table 7:** Endogeneity test.

Statistic	Statistics	Decision
Durbin (χ2)	47.298***	Endogeneity is existed (Rejection of null Hypotheses)
Wu–Hausman (f-statistics)	49.961 ***	Endogeneity is existed (Rejection of null Hypotheses)

### Diagnostic tests

#### Endogeneity test

As shown in Table 7, the Durbin and Hausman tests for endogeneity reject at a significance level of 1% the support for the null hypothesis. This indicates that the panel contains endogeneity.

#### Heteroscedasticity and autocorrelation

According to the results presented in Table 8, the Wald test for group-wise heteroscedasticity confirmed the existence of such heteroscedasticity. Since Wald group wise heteroscedasticity is present, homoscedasticity is also present. Since F-test = 207,610 is statistically significant at the 1% significance level, we reject the null hypothesis of homoscedasticity. Analysis of the panel data using the Wooldridge test revealed the presence of autocorrelation. The test results confirmed the presence of autocorrelation, as shown in Table 8. The findings presented in Table 8 refute the null hypothesis regarding the absence of first-order panel autocorrelation with a p-value of 0.000. The Wooldridge panel autocorrelation test yielded an F-statistic of 53.892. The analysis then determined whether panel data exhibited group wise heteroscedasticity by employing the Wald test.

**Table 8:** Heteroscedasticity and autocorrelation.

Test	Wald test statistic	Ho	Wooldridge test for autocorrelation	Ho
	53.892***	Rejected	207.610***	Rejected

#### Multicollinearity

VIF was used to determine the multicollinearity. Table 9 summarizes the results of the VIF analysis. According to the VIF test results, which indicated a mean value of 1.58, there was no evidence of multicollinearity.

**Table 9:** Multicollinearity (VIF results).

Variable	VIF	1/VIF
Ln (IND)	2.876	0.348
Ln (TO)	1.516	0.660
Ln (FDI)	1.426	0.701
Ln (ED)	1.366	0.732
Ln (EDS)	1.326	0.754
Ln (REC)	1.286	0.778
Mean VIF	1.633	

**Notes:** CO2 = Carbon Dioxide Emissions, IND = Industrialization, TO = Trade Openness, FDI = Foreign Direct Investment, ED = Environmental Diplomacy, EDS = Environmental Diplomacy Secure, REC = Renewable Energy Consumption.

#### GMM estimation model result

Table 10 shows the findings of the GMM estimation. At the 5% level, a t-statistic of -4.197, a p-value of 0.000, and a coefficient of -0.040 of industrialization (IND) indicate a statistically significant effect on environmental degradation. Prior researchers have reported similar findings [27,42]. Therefore, the trade openness (TO) coefficient is 0.004, with a t-statistic of 2.343 and a p-value of 0.020, indicating a statistically significant discovery at the 5% level. Prior researchers have reported similar findings [2,7,33]. Statistical evidence reveals that FDI significantly impacts environmental degradation in G20 countries, with a p-value of 0.000, a coefficient value of 0.209, and a t-statistic value of 8.86. Previous researchers found that similar results [12,21,36]. Nevertheless, environmental diplomacy (ED) is quite influential in the cause of environmental degradation. This is clear at the 99% significance level with the corresponding t-statistic value of 2.761, significant p-value value of 0.2 and the coefficient of 0.070. This has been previously observed by other researchers in the field before you, such as [13,21,33]. One of the most impactful variables for securing environmental degradation coefficient is the Environmental diplomacy secures (EDS) that has a coefficient value of -0.440 that has a t- statistic of -5.055 p-value of 0.000 and a significance level of 1%. Scholars have also recorded a similar pattern of results [21,55]. Lastly, there is environmental degradation coefficient impact value of renewable energy consumption (REC) is 0.161, t-statistic has a value of 1.881 with a p-value of 0.006 and the significance threshold of the 1% level. [1,8,13,21] also reported previous findings in this regard [49,57,58].

RETRACTED

**Table 10:** GMM estimation result.

Variable	Coefficient	Std. Error	t-Statistic	Prob.	Remarks
Ln (IND)	-0.040	0.009	-4.197	0.000	Significant ***
Ln (TO)	0.004	0.018	2.343	0.020	Significant **
Ln (FDI)	0.209	0.024	8.860	0.000	Significant ***
Ln (ED)	0.070	0.025	2.761	0.006	Significant ***
Ln (EDS)	-0.440	0.087	-5.055	0.000	Significant ***
Ln (REC)	0.161	0.0855	1.885	0.060	Significant *
C	3.091	0.369	8.381	0.000	

Notes: The variables under the study are CO2 = Carbon Dioxide Emissions, IND = Industrialization, TO = Trade Openness; FDI = Foreign Direct Investment, ED = Environmental Diplomacy; EDS = Environmental Diplomacy Secure, REC = Renewable Energy Consumption. The sign *, **, *** indicates that level of significance at 1%, **5%, and 10% respectively.

## Discussion

Industrialization exerts an important and negative influence on the environmental performance of the G20 countries. First, it paves the way for unlimited natural resource use by industries, which is a crucial factor constraining sustainable development. Industrialization has played a key role in the economic growth of the major G20 economies. Environmentally safe practices and ecologically sustainable development are becoming more significant in the contemporary world. As a result of environmental crises, most of the G20 countries are introducing new industrial rules and norms, and there are also investments in green technology and global climate change projects.

RETRACTED

On the other hand, the essence of finding a way to balance business achievement and sustainability in the environment remains an issue that could be seen as neck breaking. There is also a positive and significant dimension of openness in trade with environmental performance. However, numerous moving parts and potential benefits and costs have been depicted regarding the influence of G20 trade openness on environmental degradation. The type of traded items between these countries, technology transfer, policy coordination, and environmental rules of G20 countries are some determinants influencing the effect of trade openness on environmental pollution. Though it may worsen ecological problems, technology transfer and greener industrial practices are widely mentioned as transnational means of technology in commerce for sustainable development, which is widely promulgated. Effective legislative measures and international cooperation are needed to maintain environmental sustainability, which would weigh on the view of commerce and improve this correlation.

FDI has also significantly and positively impacted environmental performance. Consequently, the severity of environmental degradation due to foreign direct investments in G20 countries is multilayered and context dependent. The type of environmental standards, the investment that created the form, and the pre-existing laws are just a few factors that impact FDI and ecological outcomes. Foreign direct investment’s response to environmental degradation in the G20 can only have a direct impact if the various dependent aspects characterize the G20. Through FDI, policymakers can safeguard the long-term nature of environmental sustainability, including responsible investment practices, stringent environmental codes, and the transfer of technology that supports long-term goals. In the meantime, the positive relationship remains but is significantly responsible for environmental diplomacy and environmental performance. For G20 countries, environmental diplomacy is an important tool in tackling and addressing the effects of and damage to the environment. How will environmental diplomacy help in different ways in the hierarchical issues of the struggle with benefits and downsides? However, the influence of environmental diplomacy can be positive only with difficulties and hardships. Problems that squarely reduce in terms of the deadlock of international conflicts, which of opposing interests, economic stems, and certain issues intractable character as well as alliance improvement. The G20 nations are cooperative and willing to put environmental problems first so that environmental diplomacy can be successful.

RETRACTED

The negative and significant impact environmental diplomacy secure has on environmental performance is highlighted as follows: Thus, when we write, "environmental diplomacy is secure," these environmentally sound measures have stabilized and have helped reduce environmental degradation in G20 countries. Environmental diplomacy becomes effective since it helps to minimize or prevent environmental deterioration. Although secure environmental diplomacy has appreciative outcomes, acknowledging the necessity for continued costs and determined efforts to address environmental degradation’s diverse, interrelated concerns is essential. A team functioning as a truly global community adapted to honest communication and implementing agreed-upon policies and strategies is a powerful value for success. Lastly, renewable energy has demonstrated a positive and significant effect on environmental performance among G20 countries. Thus, in G20 countries, this increase in renewable energy consumption likely positively impacts environmental degradation. Notably, renewable energy sources, such as hydropower, solar, and wind energy, are environmentally friendly alternatives to conventional fossil fuels. They are ecologically preferable due to their weak planetary impact and limited greenhouse gases. While variable growth is indeed good as it could have positive environmental benefits, it is equally important to consider variables such as land use, the whole life cycle of energy technology, and the environmental implications of manufacturing and disposing of renewable energy infrastructure, which can all impact the environment. Such measures are an integrated plan wherein energy efficiency measures, conservation efforts, and sustainable natural resource management are necessary to significantly lower environmental damage.

## Conclusion

A quantitative type of research is conducted in this study, and it is about explaining variables’ correlation since we seek for the relationship of those involved: industrialization, trade openness, FDI, environmental diplomacy, security, and renewable energy consumption, against environmental degradation. Our sample utilizes panel data and includes all the countries in the G20, and our period of investigation covers the interval between 1991 and 2020. The basis for this data is the databases collected by the World Bank Global Financial Development Database (GFDD) and the IMF. The analysis of data was conducted through the two-step GMM methodology. To begin, the study examined six dimensions: industrialization, trade openness, FDI, environmental diplomacy, secure environmental diplomacy and, renewable energy is used to measure the environmental impacts in 20 countries of the G20. Thus, the current study shows that GMM estimation outcomes validated the association among autonomous factors (Justification, trade control, FDI, environmental governance, warranted environmental diplomacy, safe environmental diplomacy secure, and renewable energy) and whole effects correspondences and contaminated/damaged effects between independent and reliant factors particularly in G 20 makes. The first goal is to study variances in environmental factors and their relevance to environmental degradation. Thus, the evidence has been fulfilled as the main objective bases on environmental diplomacy, environmental diplomacy secure, and renewable energy; these factors have an adverse effect on environmental degradation. The second purpose is to tackle the influence of economic variables in the case of environmental pollution. Therefore, industrialization, trade openness, and FDI are all shown to have a key influence on environmental degradation. Lastly, these mentioned dams such as use of renewable energies, environmental diplomacy, and trade liberalization, industrialization and foreign direct investment have indubitably and complicated as well as interrelated set of effects to environmental degradation. The above factors are important in evaluation of the environmental state at a national level but also of interest to the G20 countries. A converged approach to interdependence in sustainability ecosystem and environment conservation should play out among governments, governments, corporate, and international organizations. These undertakings incorporate a range of operations namely diplomatic efforts geared at encouraging international cooperation, investing in pristine technology, ensuring effective environmental laws, and advancing sustainability. The idea that meaningful collaboration is paramount for the G20 nations and all countries to work collectively to create a future that will be sustainable in that it will represent some sort of balance between economic growth and the conservation of the natural environment is key.

RETRACTED

## Implications

### Policy implications

The results of the research have significant policy implications for the development of effective approaches to environmental degradation in the G20 countries. In this way, policymakers should target on developing and implementing wide environmental policies that incorporate diplomatic efforts, paying attention to collaborative nature. Policies should ensure sensitive balance between economic development and sustainability in the sense that the famous connection is well defined between industrial development, liberalization of trade, and the role of foreign direct investment and environmental degradation. Diplomatic negotiations and agreements need to promote clean energy sources, which are secure and renewable energies for the reduction of carbon emissions in the long term and improvement of sustainability. In addition, policymakers should focus on improving the stipulations on environment to improve on the environmental regulations both the national level and through the collaborative efforts made with other countries in terms of the environment which could be here the adverse impacts associated with the industrial activities or the foreign investments. The study focuses on the fact that a comprehensive and cohesive approach should be used by which diplomacy plays a significant role in forming policies that will benefit the welfare of both economies and the environment to the G20 countries.

### Practical implications

The practical implications of the study reveal that essential policy to actions are required within the G20 countries to ensure a balance between economic growth and environmental sustainability. The statistics duly identified the need to complement the diplomatic efforts with the mechanism of comprehensive environmental policies. Studies underline the importance of a robust framework of environmental laws that are implemented appropriately as an actionable strategic policy intervention aimed at the preservation of the environment and the economy. Such practical implications should be considered by the governments and so they should continue their way to making the paths of economic transformations greener and more sustainable, to preserve long-term resilience of the economic progress and ecological integrity.

### Limitations and future directions

Environmental diplomacy has witnessed significant contribution from other bodies including the G-20 which has had a great dominance in its conduct with other fellow countries representing the G-20 playing a big role in the formulation of international regulatory policies and engagements. On the other hand, the study conclusions may be only local because modern situation with factors of environmental, economic, and diplomatic is forever in change. This research can be followed by future country specific analyses using live data and exploration of different aspects including the impact of the non-state actors like multinational corporations and environment advocacy group on the significance of environmental diplomacy and policy outcome.

## Supporting information

S1 Data (ZIP)
